This article has been retracted.

# Value of Intensive Nursing Detail Management in Intensive Care Unit Nursing

**DOI:** 10.1155/2022/9115639

**Published:** 2022-06-22

**Authors:** Yansong Li, Lehong Zhou, Qin Wei

**Affiliations:** ^1^Nursing Department, Shiyan Maternal and Child Health Hospital, Shiyan, Hubei Province, China; ^2^Critical Care Medicine, Renmin Hospital, Hubei University of Medicine, Shiyan, Hubei 442000, China; ^3^Department of Neurosurgery, Renmin Hospital, Hubei University of Medicine, Shiyan, Hubei 442000, China

## Abstract

**Objective:**

To evaluate the value of intensive nursing detail management in intensive care unit (ICU) nursing.

**Methods:**

In this prospective study, 100 ICU patients in Shiyan Maternal and Child Health Hospital between January 2019 and March 2020 were assessed for eligibility and recruited. They were concurrently randomly assigned (1 : 1) to receive either conventional nursing (control group) or intensive nursing detail management (study group). The clinical endpoint was the nursing efficiency.

**Results:**

Intensive nursing detail management was associated with significantly higher scores in basic nursing, quality of nursing, and quality of management versus conventional nursing (*P* < 0.05). Intensive nursing detail management resulted in a significantly higher adequate nursing rate (96.00%) versus conventional nursing (74.00%) (*P* < 0.05). The patients given intensive nursing detail management had a shorter hospital stay versus those receiving conventional nursing (*P* < 0.05). Intensive nursing detail management was associated with a higher nursing satisfaction rate (74.00%) versus conventional nursing (70.00%) (*P* < 0.05).

**Conclusion:**

Intensive nursing detail management is effective and safe in ICU nursing, so it is worthy of clinical application.

## 1. Introduction

Intensive care units (ICUs) [1] provide optimal protection for critically ill patients in terms of medical resources and technology [2] and deliver the finest care, comprehensive treatment, medical and nursing integration, and early postoperative rehabilitation to obtain positive treatment outcomes [3, 4]. ICU is a form of medical organization and management that emerges with the joint development of nursing and rehabilitation, the advent of new medical equipment, and the improvement of hospital management systems [5]. The complex and rapidly changing conditions of ICU patients require timely care [6], so ICU nursing management is highly appreciated in clinical practice [7]. ICU nursing management integrates medical and nursing care [8] to ensure favorable treatment results and improve the quality of life of patients after discharge [9, 10]. Detail management is an emerging management method that highlights the details during nursing care to timely identify nursing deficiencies and thus improve the quality of care. To ensure the safety of ICU patients, improve the quality of nursing care, and avoid medical accidents, this study aimed to investigate the value of intensive nursing detail management in ICU nursing. The results are reported as follows.

## 2. Materials and Methods

### 2.1. Baseline Data

In this prospective study, 100 ICU patients in Shiyan Maternal and Child Health Hospital between January 2019 and March 2020 were assessed for eligibility and recruited. They were concurrently randomly assigned to either a control group (*n* = 50) or a study group (*n* = 50). This study was reviewed and approved by the Ethics Committee of Shiyan Maternal and Child Health hospital, SYMC01087.

### 2.2. Treatment Methods

The control group received conventional care, including condition monitoring, psychological status observation, health education, dietary guidance, and appropriate use of analgesics for pain relief [11].

The study group was given intensive nursing detail management. ① Establishment of an intensive detail management team: the team consisted of medical and nursing staff in the ICU, and the nursing staff candidates were evaluated by the head nurse and managed hierarchically in terms of their working hours, previous performance, nursing results, and nursing experience to screen out adequate nurses. ② Nursing management system: the nursing management system was developed and modified by the chief nurse of the ICU and the detail management team, and the implementation of the nursing operation, emergency plan, and specialty care was scheduled at length. ③ Preventive measures management: the team members organized the historical information on nursing management and summarized the limitations and issues of nursing to improve nursing quality. ④ Quality management of nursing: the nurses were given regular training to improve their nursing skills. The chief nurse was responsible for the assessment of the nursing work by the team members and held regular summary seminars about the nursing work, with an emphasis on assessing the professional knowledge of the nursing staff.

Patients in both groups received auricular embedding of Vaccariae Semen in the acupoints of the heart, liver, Shenmen, and Pizhixia for 30 min to calm the mind and regulate the liver and Qi. Stimulation of the auricular points induces normal orderly activation and inhibition of the reticular system of the brain, which converts the pathological sleep state to normal physiological sleep to treat insomnia.

### 2.3. Outcome Measures

1. The “Nursing Quality Evaluation Scale” developed by our hospital was used to assess the nursing quality, including three domains: basic nursing care, nursing quality, and management quality, with a total score of 100 points. The higher the score, the better the quality of nursing.
2. The quality of basic nursing and the length of hospital stay of the patients in both groups were recorded to calculate the adequate rate of nursing
3. The nursing satisfaction questionnaire (including attitude of medical staff, efficiency of medical staff, and health education quality) created by our hospital was used to assess the satisfaction of patients. It was divided into four levels, namely, highly satisfied, satisfied, less satisfied, and dissatisfied. The reliability of the scale was 0.833 and the retest consistency was 0.841.

### 2.4. Statistical Analysis

SPSS 22.0 was used for data analyses. The measurement data are expressed as (mean ± SD) and analyzed using the *t*-test. The count data are expressed as the number of cases (rate) and analyzed using the chi-square test. Differences were considered statistically significant at *P* < 0.05.

## 3. Results

### 3.1. Baseline Patient Profile

The baseline characteristics of the two groups were comparable (*P* > 0.05) (Table 1).

### 3.2. Nursing Quality

Intensive nursing detail management was associated with significantly higher basic nursing, quality of nursing, and quality of management scores (96.12 ± 5.17, 97.17 ± 3.98, and 99.45 ± 4.81) versus conventional nursing (88.43 ± 5.24, 86.54 ± 3.64, and 91.62 ± 4.23) (*P* < 0.05) (Table 2).

### 3.3. Nursing Adequacy and Length of Hospital Stay

Intensive nursing detail management resulted in a significantly higher adequate nursing rate (96.00%, including 48 cases of adequate and 2 cases of inadequate) versus conventional nursing (74.00%, including 37 cases of adequate and 13 cases of inadequate) (*P* < 0.05) (Table 3).

### 3.4. Nursing Satisfaction

The patients given intensive nursing detail management had a shorter hospital stay (11.23 ± 3.31) versus those given conventional nursing (14.61 ± 4.05) (*P* < 0.05). Intensive nursing detail management was associated with a higher nursing satisfaction rate (74.00%, including 22 (44.00%) cases of highly satisfied, 25 (50.00%) cases of satisfied, and 3 cases (6.00%) of less satisfied) versus conventional nursing (70.00%, including 12 (24.00%) cases of highly satisfied, 23 (46.00%) cases of satisfied, 9 cases (18.00%) of less satisfied, and 6 cases (12.00%) of dissatisfied) (*P* < 0.05) (Table 4).

## 4. Discussion

ICUs provide simultaneous treatment, care, and rehabilitation of critically ill patients to obtain positive lifesaving outcomes [12]. Nursing care in the intensive care unit should be scientific, effective, comprehensive, and systematic, with high requirements for nursing details [13, 14] to efficiently avoid nursing accidents and enhance patient satisfaction, thereby reducing various medical disputes [15]. Clinical practice has confirmed [16] that the application of enhanced detail management in intensive care unit nursing could achieve satisfactory nursing outcomes and significantly reduce nursing accidents in clinical settings. Detail management focuses on the quality of care [17, 18] to enhance treatment outcomes. Clinical care requires accurate nursing and dynamic monitoring of changes in the patient's condition to further improve the predictability of clinical care [19]. A previous study suggested strong demand for detail management in ICU nursing [20].

In the present study, intensive nursing detail management was associated with significantly higher basic nursing, quality of nursing, and quality of management scores, a significantly higher adequate nursing rate, and a shorter hospital stay versus conventional nursing, which may be attributed to the limited scope of routine care and the ineffectiveness of nursing issues settlement. Detail management provides standardized care, analysis of nursing defects, active communication with patients, targeted care protocols, and regular assessment of nursing staff, thereby ensuring high-quality care. Traditional Chinese medicine (TCM) can prevent sleep disorders, ICU syndrome, gastrointestinal dysfunction, oral infections, and pressure sores and psychologically help patients establish confidence against diseases to enhance treatment compliance. Moreover, TCM preparations are relatively inexpensive with few side effects and can save substantial medical resources and costs. Patients in ICU experience dysfunction of internal organs and deficiency of Qi and blood, and prolonged bed-rest pressure results in the formation of local ulcers and necrosis, which aggravates patients' pain. Auricular compression or embedding can prevent pressure sores by using the large and small fissure muscles of the palm to massage at the patient's bony prominence twice a day to reduce swelling and pain, activate blood circulation, and prevent pressure sores.

Patients in ICU need to be bedridden for a long time and cannot move independently, which predisposes them to complications. After the vital signs of the critically ill patient are relatively stable, the lower limbs are kept elevated to promote venous blood return and facilitate limb rehabilitation exercises. The patients are given limb massage to prevent muscle atrophy and joint deformation. The nursing staff assists the patient to perform early passive or active movement of the quadriceps in bed and to perform dorsiflexion and plantarflexion of the ankle joint for about 30 min daily. If the patients can perform these movements, they are gradually allowed to move the ankle joint independently, carry out foot stirrups and straight leg raises to dorsiflex the foot, and then forcefully tense the knee joint, and a top-down and rhythmic compression of the gastrocnemius muscle was performed [3]. The massage and functional activities prevent the formation of venous thrombosis in the lower extremities while promoting the recovery of ribbed lower extremity function.

Moreover, intensive nursing detail management resulted in a higher nursing satisfaction rate versus conventional nursing, which is consistent with the results of the previous research. Detail management optimizes the nursing process, strengthens the motivation of nursing staff, and reduces nurse-patient disputes due to inappropriate handling of details or poor communication, leading to improved patient satisfaction. The above results of the present study suggested the promising nursing efficiency of intensive nursing detail management for ICU patients.

## 5. Conclusion

Intensive detail management significantly reduces nursing disputes due to nursing errors and nursing defects in clinical practice, and its application to intensive care unit nursing shows pronounced nursing benefits and high safety, so it is worthy of clinical application.

## Figures and Tables

**Table 1:** Comparison of baseline data ($\bar{\text{x}}$ ± *s*).

Groups	*n*	Gender		Mean age	Mean disease duration
		Male	Female		
Study group	50	28	22	52.88 ± 7.61	2.18 ± 0.94
Control group	50	26	24	53.09 ± 8.21	2.25 ± 0.81
*t*/*X*^2^ value			2.365	0.384	0.785
*P* value			0.532	0.723	0.451

**Table 2:** Comparison of nursing quality ($\bar{\text{x}}$ ± *s*).

Groups	*n*	Basic nursing	Quality of nursing	Quality of management
Study group	50	96.12 ± 5.17	97.17 ± 3.98	99.45 ± 4.81
Control group	50	88.43 ± 5.24	86.54 ± 3.64	91.62 ± 4.23
*t* value	—	5.617	4.911	6.171
*P* value	—	<0.001	<0.001	<0.001

**Table 3:** Comparison of nursing adequacy and length of hospital stay ($\bar{\text{x}}$ ± *s*, %).

Groups	*n*	Adequate	Inadequate	Hospital stays (d)
Study group	50	48 (96.00)	2 (4.00)	11.23 ± 3.31
Control group	50	37 (74.00)	13 (26.00)	14.61 ± 4.05
*t*/*X*^2^	—	5.423		4.682
*P*	—	0.028		0.001

**Table 4:** Comparison of nursing satisfaction (%).

Groups	*n*	Highly satisfied	Satisfied	Less satisfied	Dissatisfied	Satisfaction rate
Study group	50	22 (44.00)	25 (50.00)	3 (6.00)	0 (0.00)	47 (94.00)
Control group	50	12 (24.00)	23 (46.00)	9 (18.00)	6 (12.00)	35 (70.00)
*X* ^2^	—	5.585				
*P* value	—	<0.001				

## Data Availability

No data were used to support this study.
